This article has been retracted.

# Systematic Understanding of the Mechanism of Baicalin against Gastric Cancer Using Transcriptome Analysis

**DOI:** 10.1155/2021/5521058

**Published:** 2021-07-19

**Authors:** Wenqu Zhou, Mi Gao, Chunxiao Liang, Biting Lin, Qinghua Wu, Ruikun Chen, Xiaoxiao Xiong, Xing Chen, Shijie Wang, Liting Wu, Yiling Wu, Haiqing Li, Xin Fu, Wei Hong

**Affiliations:** ^1^GMU-GIBH Joint School of Life Sciences, Guangzhou Medical University, Guangzhou, Guangdong, China; ^2^State Key Laboratory of Respiratory Disease, National Clinical Research Center for Respiratory Disease, Guangzhou Institute of Respiratory Health, The First Affiliated Hospital of Guangzhou Medical University, Guangzhou Guangdong, China; ^3^Department of Thoracic Medicine, Shenzhen Second People's Hospital, The First Affiliated Hospital of Shenzhen University, Shenzhen, Guangdong, China; ^4^The Third Clinical School of Guangzhou Medical University, Guangzhou Guangdong, China

## Abstract

**Background:**

Gastric cancer (GC) is the most common type of cancer. It is highly malignant and is characterized by rapid and uncontrolled growth. The antitumour activity of Baicalin was studied in multiple cancers. However, its mechanism of action has not been fully elucidated. We provided a systematic understanding of the mechanism of action of baicalin against GC using a transcriptome analysis of RNA-seq.

**Methods:**

Human GC cells (SGC-7901) were exposed to 200 *μ*g/ml baicalin for 24 h. RNA-seq with a transcriptome, Gene Ontology (GO), and Kyoto Encyclopedia of Genes and Genomes (KEGG) enrichment analyses were used to identify the antitumour effects of baicalin on SGC-7901 cells in vitro. A protein-protein interaction (PPI) network of differentially expressed genes (DEGs) was constructed. A competitive endogenous RNA (ceRNA) network was constructed and further analysed after validation using qRT-PCR.

**Results:**

A total of 68 lncRNAs, 20 miRNAs, and 1648 mRNAs were differentially expressed in baicalin-treated SGC-7901 GC cells. Three lncRNAs, 6 miRNAs, and 7 mRNAs were included in the ceRNA regulatory network. GO analysis revealed that the main DEGs were involved in the biological processes of the cell cycle and cell death. KEGG pathway analysis further suggested that the p53 signalling pathway was involved in the baicalin-induced antitumour effect on SGC-7901 cells. Further confirmation using qPCR indicated that baicalin induced an antitumour effect on SGC-7901 cells, which is consistent with the results of the sequencing data.

**Conclusions:**

In summary, the mechanism of baicalin against GC involves multiple targets and signalling pathways. These results provide new insight into the antitumour mechanism of baicalin and help the development of new strategies to cure GC.

## 1. Introduction

Gastric cancer (GC) is one of the leading prevalent type of malignancies and has the second highest cancer-related mortality rate in China [1]. The distant migration and invasion of GC cells are the main causes of mortality from GC [2]. Most patients have metastases at the time of diagnosis, and the 5-year survival rates is extremely low [3]. Patients who receive advanced treatment for GC, including surgery combined with radiotherapy, chemotherapy, and targeted therapy, still experience treatment failure and have poor outcomes, such as inadequate therapeutic effects, high toxicity, recurrence, and metastasis [4]. Therefore, it is of urgency and importance to identify an effective treatment for GC.

Risk factors for GC (or stomach cancer) include diet, lifestyle, and family history, of which diet has been considered to be the primary risk factor. The consumption of food preserved by salting, smoking, or pickling can contribute to the development of GC, although these methods have preservation have commonly been replaced by refrigeration. However, shift in the method of food preservation has resulted in other food safety concern. Food safety is one of the leading issues for human beings and public health, and there are two major concerns: food poisoning and food spoilage. Food poisoning is commonly caused by different pathogens, including *Escherichia coli*, *Salmonella*, *Staphylococcus aureus*, *Listeria monocytogenes*, *Vibrio parahaemolyticus*, and *Pseudomonas aeruginosa* [5–10]. With regard to food spoilage, *Lactobacillus* and *Bacillus* are major causes, and their “hard to culture” or “viable but unculturable” status has compounded the problem [11–14]. The critical role of the pathogen *Helicobacter pylori* in the development of GC has been well documented [15]. However, the colonization, growth, persistence, and life cycle of microorganisms does not occur in isolation; rather, these microorganisms interact with each other. For example, antimicrobial resistance in such pathogens, biofilm formation, and polymicrobial interactions, further complicate problem [16–23]. Since diet and food safety play an important roles in the development of GC, the future preventive measures or therapies could involve food safety and diet considerations. One important example is natural products or food additives. Natural products have recently received attention with regard to the search for of novel anticancer therapeutic agents because these products have long been used as alternative remedies for a variety of diseases, including cancer, with relatively few side effects. Baicalin is the predominant flavonoid isolated from the roots of *Scutellaria baicalensis* Georgi (Huang Qin), and it exhibits various pharmacological activities, including antioxidative, antiviral, anti-inflammatory, and anticancer activities [24]. Significant antitumour effects of baicalin were observed against lung cancer [25], colon cancer [26], pancreatic cancer [27], breast cancer [28], and nasopharyngeal carcinoma [29]. However, the molecular mechanisms underlying the contribution of baicalin to cancer treatment remain elusive. Our previous study reported that baicalin induced apoptosis in GC cells, but the underlying molecular mechanisms were not clear. Transcriptome profiling is an important tool for understanding the possible mechanisms at the transcriptional level. High-throughput RNA sequencing (RNA-seq) is one of the most popular technologies used for genome-wide transcriptome profiling.

Noncoding RNAs (ncRNAs) are RNA transcripts that do not encode proteins and are classified as small ncRNAs (sncRNAs, 18~200 nt) and long ncRNAs (lncRNAs, >200 nt). There are different kinds of sncRNAs, such as microRNAs (miRNAs). ncRNAs are involved in most cellular functions, such as proliferation, apoptosis, endothelial-to-mesenchymal transition (EMT), autophagy, and cell cycle control. Multiple ncRNAs act as oncogenes or tumour suppressor genes during carcinogenesis and serve as diagnostic and prognostic markers in cancer patients after certain therapies [30]. Emerging evidence has demonstrated that lncRNAs function as molecular sponges for miRNA via their miRNA response elements (MREs) and influence the translation inhibition or mRNA degradation of the transcript on the targets by the respective miRNAs, which was proposed as the competing endogenous RNA (ceRNA) hypothesis [31]. Various elements of this complex crosstalk of the ceRNA network are involved in GC. lncRNA MALAT1 modulates oxaliplatin resistance in gastric cancer by sponging miR-22-3p [32]. lncRNA MALAT1 potentiates autophagy-associated cisplatin resistance by regulating the microRNA-30b/autophagy-related gene 5 axis in GC [33]. lncRNA LINC01234 functions as a competing endogenous RNA to regulate CBFB expression by sponging miR-204-5p in GC [34]. However, few studies have investigated the ceRNA mechanisms of lncRNAs in baicalin-treated cancer are rare.

The present study had characterized the global gene expression profiles of the baicalin-treated SGC-7901 GC cells using RNA-seq. A reference genome analysis of the transcriptome was performed, and the profile of differentially expressed genes (DEGs), their functions, and the mechanisms involved in the antitumour effects of baicalin were investigated. Our findings help reveal the complex biological processes and molecular mechanisms mediating the antitumour effects of baicalin and highlight that ncRNAs may act as potential biomarkers and/or therapeutic targets of GC.

## 2. Materials and Methods

### 2.1. Cell Culture

Human GC cells (SGC-7901) were obtained from Guangzhou Medical University, which sourced the cell line from the American Type Culture Collection (Manassas, VA, USA). SGC-7901 cells were cultured in the recommended medium supplemented with 10% foetal bovine serum (FBS; Gibco, USA) at 37°C in a humidified atmosphere with 5% CO_2_. Cell passage was performed every 2-3 days. Baicalin (purity, ≥95%, Sigma-Aldrich, St. Louis, MO, USA) was dissolved in dimethyl sulfoxide (DMSO) in a 0.4 g/ml stock solution. The same volume of DMSO with a final concentration of 0.1% was used as a negative control. SGC-7901 cells were stimulated with baicalin (200 *μ*g/ml) for 24 h as in our previous study.

### 2.2. RNA Preparation and RNA Sequencing

Total RNA was isolated using the miRNeasy Mini Kit (Qiagen) according to the manufacturer's protocols and then treated with RNase-Free DNase to remove residual genomic DNA contamination. The quality and quantity of the RNA used to generate the RNA sequencing libraries were assessed using an Agilent 2100 Bioanalyzer (Agilent Technologies). The RNA-seq library was prepared from 20 ng of total RNA. RNA sequencing was performed with a Hiseq 2500 system (Illumina, Inc., San Diego, CA, USA).

### 2.3. Read Mapping and Genome Annotation

The raw reads were evaluated and cleaned using the online software FastQC to remove ligation sequences, low-quality sequences, and repeats. After filtering, the useful reads were mapped to the human genome version GRCh37 using HISAT2 software. StringTie software was used to assemble the transcripts, and the Perl script was used to screen for known lncRNAs. We obtained the resulting known lncRNAs and used CPC and PFAM software to predict the novel lncRNAs. We also used the reads that were mapped to the genome to perform additional alignments using different software programs, including NCGB, Rfam, and Hairpin to classify the types of reads. We obtained the resultant known miRNAs and used the unknown reads to predict the novel miRNAs.

### 2.4. Analysis of DEGs

The quantitative analysis of lncRNAs and mRNAs was performed using the R package Ballgown, and the lncRNA target mRNAs were predicted. All known miRNAs and novel miRNAs were used to calculate expression levels by performing analysis of variance (ANOVA) on the transcript per million (TPM) count. After obtaining the differential expression of the targeted mRNA and miRNA reads, we predicted the targets and performed an enrichment analysis. GO (http://www.geneontology.org) and KEGG (http://www.genome.jp/kegg) analyses were performed for the differentially expressed miRNA- (DEmiRNA-) associated genes. A *P* value < 0.05 was considered significant. The top 20 significant pathways involving the upregulated and downregulated miRNAs were chosen to construct the pathway relation network, which was based on the interaction data in KEGG. The pathway relation network was used to identify the regulatory effect of these pathways.

### 2.5. Protein-Protein Interaction (PPI) Network

The PPI network of DEGs was constructed and visualized using Cytoscape software (version 3.6.1; https://www.cytoscape.org) based on the interaction data from the Search Tool for the Retrieval of Interacting Genes (version 10.0; https://www.string-db.org/) database.

### 2.6. Constructing the ceRNA Network

The lncRNA-miRNA-mRNA ceRNA network was based on the ceRNA hypothesis that ceRNAs can coregulate each other by competing for shared MREs. To construct the network, lncRNA-miRNA interactions retrieved from miRanda (http://www.microrna.org/microrna/home.do), miRTarBase (http://mirtarbase.mbc.nctu.edu.tw/), and TargetScan (http://www.targetscan.org/) were used to predict the target genes of the miRNAs. Then, the differentially expressed lncRNAs, miRNAs, and mRNAs with false discovery rate (FDR) < 1%, absolute log 2‐fold change > 2, and *P* < 0.05 were retained and used to establish the ceRNA network. Cytoscape 3.6.1 was used to construct and visualize the network.

### 2.7. Quantitative Real-Time PCR (qRT-PCR) Validation

To further improve the reliability of the ceRNA network, we selected some of the key RNAs in the ceRNA network and used qRT-PCR for validation. RNA samples from SGC-7901 cells treated with baicalin (200 *μ*g/ml) were collected. Total RNA was extracted using the TRIzol reagent (Invitrogen, CA, USA). cDNA was synthesized from 1.0 *μ*g of total RNA using the PrimeScript RT™ Reagent Kit according to the manufacturer's instructions (TaKaRa, Japan). qRT-PCR was performed using SYBR Premix Ex Taq™ (TaKaRa) and the Step-One Fast Real-Time PCR system on the CFX Connect™ Real-Time PCR system (Bio-Rad, USA). To quantify the results, the relative expression levels were calculated using the 2^−ΔΔCt^ method. The PCR conditions were 2 min at 95°C, 40 cycles at 95°C for 5 s, and 60°C for 34 s. The data represent the means of three experiments. The primer sequences are shown in Table 1.

### 2.8. Statistical Analysis

Data are expressed as the means ± SD. All statistical analyses were performed using SPSS 23.0 (SPSS, Chicago, IL, United States). A *P* value < 0.05 was considered significant.

## 3. Results

### 3.1. Differentially Expressed lncRNAs, miRNAs, and mRNAs

The present study screened for differentially expressed lncRNAs (DElncRNAs), differentially expressed miRNAs (DEmiRNAs), and differentially expressed mRNAs (DEmRNAs) using RNA-Seq analysis. Untreated and baicalin-treated SGC-7901 GC cells were selected for the gene expression assay. Genes with a fold change in expression > 2.0 and *P* < 0.05 between untreated and baicalin-treated samples were identified as differentially expressed. Our project detected 68 lncRNAs, 20 miRNAs, and 1648 mRNAs. Hierarchical clustering and volcano plots showed the DElncRNAs, DEmiRNAs, and DEmRNAs between untreated and baicalin-treated SGC-7901 cells (Figure 1). There were 68 DElncRNAs (32 upregulated and 36 downregulated), 20 DEmiRNAs (15 upregulated and 5 downregulated), and 1648 DEmRNAs (959 upregulated and 689 downregulated) in the baicalin-treated cells compared to the untreated cells.

### 3.2. GO and KEGG Enrichment Analyses of DEmRNAs

GO analysis covers three domains: biological process (BP), cellular component (CC), and molecular function (MF). For further insight into the major biological function of the dysregulated genes, GO and KEGG analyses were performed. GO analysis showed that the DEGs were mainly involved in cell death and cell cycle, the intracellular and extracellular part, transferase activity, and transcription factor binding (Figure 2(a)). KEGG pathway analysis indicated that the DEGs were strongly associated with mismatch repair, DNA replication, nucleotide excision repair, the p53 signalling pathway, and oxidative phosphorylation (Figure 2(b)).

### 3.3. Construction of a PPI Network from the DEGs

Protein network visualization plays an important role in the efficient and intuitive analysis of protein network characteristics and the investigation of the behaviour of the cell machinery [35]. We used the online database STRING and Cytoscape software to construct a PPI network of the DEGs. The network contained 61 DEGs. Genes with red triangles were upregulated, and genes with blue triangles were downregulated in SGC-7901 cells treated with baicalin compared to the control group (Figure 3).

### 3.4. Construction of the ceRNA Network

To improve our understanding of the role of DElncRNAs in SGC-7901 cells treated with baicalin, a ceRNA network was constructed. As shown in Figure 4, the ceRNA network was composed of 3 lncRNAs (ENST00000526897, ENST00000582141, and ENST00000567093), 6 miRNAs (hsa-miR-5001-3p, hsa-miR-6837-3p, hsa-miR-6511a-5p, hsa-miR-6511b-5p, hsa-miR-214-3p, and hsa-miR-10396a-5p), and 7 mRNAs (CARD14, AHRR, LARP4B, EXOC6B, ACACA, FAM179A, and MDM2).

### 3.5. Validation of Representative lncRNAs, miRNAs, and mRNAs in ceRNA

Three lncRNAs, 6 miRNAs, and 3 mRNAs from the ceRNA network were chosen for verification using qRT-PCR. The qRT-PCR assay showed that the expression levels of ENST00000526897, ENST00000567093, and ENST00000582141 were downregulated in SGC-7901 cells treated with baicalin compared to the control group. The expression levels of hsa-miR-214-3p, hsa-miR-5001-3p, hsa-miR-6511b-5p, hsa-miR-6837-3p, hsa-miR-6511a-5p, and hsa-miR-10396a-5p were upregulated, and the expression levels of 3 target mRNAs, namely CARD14, FAM179A, and AHRR, were downregulated in SGC-7901 cells treated with baicalin compared to the control cells (Figure 5). The results were consistent with the sequencing data.

## 4. Discussion

GC is a malignancy with high morbidity and mortality, and it is the third leading cause of cancer-related mortality worldwide. Therefore, the need for new and effective anti-GC drug treatments is urgent. Baicalin is the major bioactive flavone derived from the root of *Scutellaria baicalensis*, which is commonly used in traditional Chinese medicine. Accumulating evidence shows that baicalin exerts remarkable bioactivities, including anti-oxidative and anti-inflammatory activities, with little toxicity to normal tissues. The anticancer function of baicalin in various cancers has recently been discovered, and baicalin occupies an important position in clinical practice [36]. However, the specific mechanisms underlying the contribution of baicalin to cancer treatment are not known. The present study for the first time meaningful evidence regarding DElncRNAs, DEmiRNAs, and DEmRNAs in SGC-7901 cells following the administration of baicalin in vitro using the high-throughput RNA-seq technique. We compared, predicted, and integrated differentially expressed RNAs to construct a differentially expressed lncRNA-miRNA-mRNA ceRNA network that elucidated the roles of baicalin in GC. The results of this study further our understanding of the molecular mechanism underlying the effects of baicalin treatment on GC. GC is one of the most invasive malignant tumours, and a deeper understanding its molecular pathogenesis is urgently needed.

Our findings had identified 68 DElncRNAs, 20 DEmiRNAs, and 1648 DEmRNAs in baicalin-treated SGC-7901 GC cells, and 3 lncRNAs (ENST00000526897, ENST00000582141, and ENST00000567093), 6 miRNAs (hsa-miR-5001-3p, hsa-miR-6837-3p, hsa-miR-6511a-5p, hsa-miR-6511b-5p, hsa-miR-214-3p, and hsa-miR-10396a-5p), and 7 mRNAs (CARD14, AHRR, LARP4B, EXOC6B, ACACA, FAM179A, and MDM2) were included in the ceRNA regulatory network after additional analysis. To further investigate the cellular mechanisms involved in the roles played by baicalin in the treatment of GC, GO analysis of the DEmRNAs was performed. GO analysis indicated that DEmRNAs were primarily enriched in the biological processes (BPs) of cell death and cell cycle, intracellular and intracellular part of cellular components (CCs), and transferase activity and transcription factor binding MFs, which are associated with gene mutations and the apoptosis of GC cells. These findings are consistent with current GC research. We also demonstrated that the results were enriched in mismatch repair, DNA replication, nucleotide excision repair, the p53 signalling pathway, and oxidative phosphorylation using KEGG pathway analysis, and these pathways are closely related to the progression of cancer. Taken together, these findings indicate that the results of RNA-seq in cancer are relatively accurate.

De-ceRNAs are closely related to the occurrence, development, and prognosis of cancer. Previous studies demonstrated that ceRNAs affected the proliferation, growth, differentiation, apoptosis, and other biological behaviours of cancer cells. ceRNAs, also known as miRNA “decoys” or miRNA “sponges,” are RNA transcripts that compete for binding to the same miRNA via base pairing with MREs, which subsequently enables a reduction in the amount of miRNAs that are available to target mRNAs [37].

NcRNAs are a large class of RNA molecules that do not encode proteins but play regulatory effects. LncRNA is a generic term for a class of RNA molecules with lengths > 200 nucleotides, and currently constitutes one of the most active fields of study in molecular biology. lncRNAs regulate the gene expression of tumour cells via multiple modes of action and are widely involved in the occurrence and metastasis of tumours [38]. LncRNAs play an important role in the development of cancer, but the functional roles of only a few have been well characterized. The present study identified 3 lncRNAs (ENST00000526897, ENST00000582141, and ENST00000567093) in the ceRNA network. ENST00000567093 is involved in the molecular pathogenesis of hypertrophic cardiomyopathy (HCM) and can be used as a candidate diagnostic biomarker or potential therapeutic target for HCM. However, ENST00000526897 and ENST00000582141 have rarely been studied.

MiRNAs are a class of sncRNAs with a length of 20-24 nucleotides that can regulate gene expression at the posttranscriptional level. Emerging evidence shows that specific miRNAs play important roles in tumour progression and function as tumour suppressor genes or oncogenes [39]. Increasing numbers of studies have shown that abnormal miRNA expression is involved in many types of cancer [40], including GC. Therefore, miRNAs are potentially useful biomarkers in clinical diagnosis as a key factor in signal cascades and may become targets and tools for cancer treatment development. hsa-miR-214-3p [41], sa-miR-5001-3p [42], and hsa-miR-6511b-5p [43] exert regulatory roles in tumour progression.

miRNAs regulate gene expression mainly by inducing targeted mRNA degradation. The present study identified 7 mRNAs that were associated with baicalin-treated SGC-7901 cells in the ceRNA network. Caspase recruitment domain family member 14 (CARD14) is a member of the CARD family of proteins that regulates cell proliferation and migration in breast cancer cells, and it is a novel potential therapeutic target in breast cancer [44]. FAM179A is closely related to lung cancer [45, 46]. Acetyl-CoA carboxylase A (ACACA), which is the crucial rate-limiting enzyme in the fatty acid biosynthesis pathway that catalyses the conversion of acetyl-CoA to malonyl-CoA, is the first step in fatty acid biosynthesis, and it occurs early in tumour progression [47, 48].

The selected RNAs included in the ceRNA network were verified using qRT-PCR to confirm the reliability and validity of the above bioinformatics results. The verified expression levels of 12 RNAs were consistent with the sequencing results, which indicates the high degree of confidence in this network. We verified the expression of the independent RNAs, and the results supported our findings and provided a better understanding of lncRNA-related ceRNAs and their important role in baicalin-treated SGC-7901 cells.

## 5. Conclusions

In summary, the present study investigated lncRNA-mediated ceRNA interactions using lncRNA, miRNA, and mRNA expression profiles in baicalin-treated SGC-7901 cells. The results provide novel insights into the mechanism underlying the pathogenesis and development of GC. This study further provides new prognostic biomarkers and therapeutic targets that can be used to guide the treatment and in-depth investigation of GC.

## Figures and Tables

**Figure 1:** Identification of DElncRNAs, DEmiRNAs, and DEmRNAs in gastric cancer. Hierarchical clustering of DElncRNAs (a), DEmiRNAs (b), and DEmRNAs (c) between untreated and baicalin-treated SGC-7901 GC cells. Red color indicates upregulation, and green color indicates downregulation. Volcano plot showing DElncRNAs (d), DEmiRNAs (e), and DEmRNAs (f) between untreated and baicalin-treated SGC-7901.

**Figure 2:** GO and KEGG pathway enrichment analysis of target genes. (a) GO enrichment of mRNAs interacting with lncRNAs. Points of different shapes represent BPs, CCs, and MFs from the GO analysis, and the bar plot shows the number of genes enriched in the GO function. (b) Histogram of KEGG pathway enrichment in baicalin-treated SGC-7901 cells. The size of the dots represents the number of genes annotated in the pathway, and the color of the dots represents the corrected *P* value of the hypergeometric test.

**Figure 3:** Protein-protein interaction (PPI) network analysis of DEGs. Red triangles represent genes that are upregulated, and blue triangles represent genes that are downregulated.

**Figure 4:** ceRNA network analysis of DElncRNAs, DEmiRNAs, and DEmRNAs in baicalin-treated SGC-7901 cells compared to those in the control group. In the network, red circles represent lncRNAs, blue rectangles represent miRNAs, and green triangles represent.

**Figure 5:** The qRT-PCR results of 3 DElncRNAs, 6 DEmiRNAs, and 3 DEmRNAs were compared with the sequencing results. The vertical axis represents the mean fold change (FC) (log2 scale) of each RNA measured by RNA sequencing or qRT-PCR. ^∗^*P* < 0.05, ^∗∗^*P* < 0.01, compared with the control (*n* = 3).

**Table 1:** Primer sequences used for qRT-PCR analysis.

Gene name	Primer sequence (5′-3′)
*lncRNA*	
ENST00000526897	
Forward	AGGCTGCTGTCTCCCACAAGAAT
Reverse	AAGCTGGAGCAGCGGATTGC
ENST00000567093	
Forward	TGGAGAGTGTCACCCCATCT
Reverse	TTTGGTTAGGTAGGCGGCAG
ENST00000582141	
Forward	CCTGTTGAGTTTGGTGGGGA
Reverse	CAAATCTGACACGCAACCCC
GAPDH	
Forward	CAGCCTCAAGATCATCAGCA
Reverse	ACAGTCTTCTGGGTGGCAGT
*miRNA*	
hsa-miR-214-3p	
Forward	GCGACAGCAGGCACAGACA
Reverse	AGTGCAGGGTCCGAGGTATT
RT	GTCGTATCCAGTGCAGGGTCCGAGGTATTCGCACTGGATACGACACTGCC
hsa-miR-5001-3p	
Forward	GCGTTCTGCCTCTGTCCAG
Reverse	AGTGCAGGGTCCGAGGTATT
RT	GTCGTATCCAGTGCAGGGTCCGAGGTATTCGCACTGGATACGACAAGGAC
hsa-miR-6511b-5p	
Forward	CTGCAGGCAGAAGTGGGG
Reverse	AGTGCAGGGTCCGAGGTATT
RT	GTCGTATCCAGTGCAGGGTCCGAGGTATTCGCACTGGATACGACTGTCAG
hsa-miR-6837-3p	
Forward	GCCGAGCCTTCACTGTGACTCTG
Reverse	CTCAACTGGTGTCGTGGA
RT	CTCAACTGGTGTCGTGGAGTCGGCAATTCAGTTGAGCCTGCAGC
hsa-miR-6511a-5p	
Forward	GCCGAGCTGCAGGCAGAAGTG
Reverse	CTCAACTGGTGTCGTGGA
RT	CTCAACTGGTGTCGTGGAGTCGGCAATTCAGTTGAGCTGTCAGCC
hsa-miR-10396a-5p	
Forward	GCGGGCGGGGCTCGGA
Reverse	AGTGCAGGGTCCGAGGTATT
RT	GTCGTATCCAGTGCAGGGTCCGAGGTATTCGCACTGGATACGACCCCGGC
U6	
Forward	CTCGCTTCGGCAGCACA
Reverse	AACGCTTCACGAATTTGCGT
*mRNA*	
CARD14	
Forward	ACATGGTTTCCTCCTGTGAGCTGG
Reverse	TTCTCATTCTCCTCCTTCAGGCGG
FAM179A	
Forward	AACAACGAGGAACCGTCACAGCT
Reverse	TCCTGGGGTGACCATTCCTTG
AHRR	
Forward	CGGGTGTGCCTGAGCC
Reverse	CACCCGGAGGTAACTGACAC

## Data Availability

The datasets used and/or analyzed during the current study are available from the corresponding author on reasonable request.
